# Evaluation of Angiogenesis and Pathological Classification of Extrahepatic Cholangiocarcinoma by Dynamic MR Imaging for E-Healthcare

This article has been retracted.

**DOI:** 10.1155/2021/8666498

**Published:** 2021-10-11

**Authors:** Jinyun Tan, Xijun Sun, Shaoyu Wang, Baoqin Ma, Zhaohui Chen, Yaowei Shi, Li Zhang, Mohd Asif Shah

**Affiliations:** ^1^Department of Hepatobiliary and Pancreatic Surgery, Lanzhou Second People's Hospital, Lanzhou, Gansu Province, China; ^2^Department of Medical Imaging, The Second People's Hospital of Lanzhou, Lanzhou, Gansu Province, China; ^3^MR Scientific Marketing,Siemens Healthineers, Shanghai, China; ^4^Bakhtar University, Kabul, Afghanistan

## Abstract

For staging cholangiocarcinoma and determining respectability, MR is an accurate noninvasive method which provides size of tumor and vascular patency information. Dynamic contrast-enhanced magnetic resonance imaging (DCE-MRI) is a noninvasive inspection method for evaluating the vascular structure and functional characteristics of tumor tissue. However, some limitations should be noted about the technology. At present, the technology cannot be used alone, which is just an assisted method during the conventional MRI examination. 50 ECC patients, admitted to Indira Gandhi Medical College and Hospital between 2016 and 2019, were selected as research subjects. They were classified pathologically according to the Steiner classification system. After image processing, regions of interest (ROIs) were selected from the image to measure the rate constant (Kep), extravascular space volume fraction (Ve), and tissue volume transfer constant (Ktrans). There were 15 cases with highly differentiated carcinoma, 23 cases with moderately differentiated carcinoma, and 12 cases with lowly differentiated carcinoma. Non-VEGF expression was noted in 21 cases, with low expression noted in 15 cases, moderate expression noted in 14 cases, and no high expression case noted. The relevant parameters in the dynamic MRI image can quantitatively reflect the angiogenesis and pathological classification of ECC, which is suggested in the clinical treatment of ECC. The Ktrans, Kep, and Ve values of the ECC patients were all not associated with the pathological classification, with no significant difference (*P* < 0.05). Besides, due to the fact that the patient cannot completely hold his breath, the air leak reduces the image quality.

## 1. Introduction

The conventional MRI results lack objective evaluation indexes, making it difficult to observe the subtle changes in the disease tissue. Dynamic contrast-enhanced magnetic resonance imaging (DCE-MRI) is a noninvasive inspection method for evaluating the vascular structure and functional characteristics of tumor tissue. Through intravenous injection of small molecule contrast agent, the circulation in the blood vessel and its pharmacokinetic characteristics are recorded [1]. It is mainly used in the diagnosis of benign and malignant lesions and tumor radiotherapy and chemotherapy effect monitoring. The detection effect is especially obvious for tumor tissues with better differentiation.

ECC is the malignant tumor that originates from the confluence of the left and right hepatic ducts to the common bile duct lower end, usually with cancers located in the ampulla and papilla excluded [2], but hilar cholangiocarcinoma accounts for more than 50%, with malignant obstructive jaundice as the main clinical symptom. The disease is characterized by slow tumor growth and advanced metastasis, mainly local lymphatic metastasis. Most patients die of various complications caused by biliary obstruction instead of tumor metastasis, and surgical resection is the main treatment method [3].

The incidence of ECC has gradually increased. Pathological studies have found that most patients with ECC have better pancreatic cancer tissues differentiation, and the differentiation of pancreatic cancer cells is nearly normal. Therefore, no obvious tumor markers can be detected in the serum, which inhibits the accurate diagnosis of the disease [2].

Between the decades of 6th and 7th, cholangiocarcinoma is common in men as compared to women. There is a tumor development at a younger age led by the presence of the choledochal cyst Caroli disease hepatolithiasis [4–6]. The mortality from hepatic failure and cholangiocarcinoma is reduced resulted by the liver transplantation [7–10]. The cholangiocarcinoma and the histologic stage of PSC may be simultaneously diagnosed. The cholangiocarcinoma is higher associated with ulcerative colitis UC as suggested by the experts [11, 12].

The cholangiocarcinomas are anatomically classified into three groups. The anatomic distribution of the tumor is correlated by these categories and preferred treatment is implied. The classification of cholangiocarcinoma is shown in Figure 1.

The cholangiocarcinoma growth has been described macroscopically; first is that mass-forming results in the liver parenchyma definite mass, as shown in Figure 2.

Second infiltrating type results in peripheral ducts dilatation which is either diffusely infiltrating or nodular, as shown in Figure 3.

The last one is the polypoidal growth type in which the lumen of the bile duct is proliferated, as shown in Figure 4. More than one growth type encompassed by the combined cholangiocarcinoma encompasses is more commonly seen with intrahepatic tumors.

The squamous cell carcinoma, small cell carcinoma, and undifferentiated types are included in tumor types [13–15]. There is variation of tumor grades from well-differentiated to undifferentiated. The clusters of cells are consisted in the most of the tumors which are surrounded by the desmoplastic stroma [16]. The reactive tissue and well-differentiated cholangiocarcinoma are difficult to distinguish. As a source for metastases, a primary adenocarcinoma should be omitted when intrahepatic cholangiocarcinoma is considered [17, 18].

Tumor blood vessels not only provide oxygen and nutrients for cell metabolism during tumor growth but are also responsible for removing waste generated by cell metabolism, serving tumor infiltration and metastasis. The new blood vessels are continuously generated during metastasis, and the increasing number of blood vessels generated indicates faster tumor growth. VEGF exerts strong effect on inducing tumor angiogenesis, and MVD is usually used to evaluate tumor angiogenesis. The VEGF and MVD values are both determined by invasive examination, and the detection is susceptible to the sample site, resulting in inaccurate measurement results [19].

Therefore, in this study, DCE-MRI was adopted to evaluate angiogenesis and pathological classification of ECC patients.

Contribution: attention given to the application of dynamic MR imaging in the evaluation of angiogenesis and the pathological classification of extrahepatic cholangiocarcinoma (ECC) patients. Therefore, in this study, DCE-MRI was adopted to evaluate angiogenesis and pathological classification of ECC patients.

1. 50 ECC patients, admitted to Indira Gandhi Medical College and Hospital between 2016 and 2019, were selected and classified pathologically according to the Steiner classification system.
2. To observe the expression of VEGF determined through immunohistochemical staining, and the MVD is determined by CD34 staining. All patients underwent the dynamic MR imaging examination.
3. After image processing, three regions of interest (ROIs) were selected from the image to measure the rate constant (Kep), extravascular extracellular space volume fraction (Ve), and tissue volume transfer constant (Ktrans).

The organization of the paper is as follows. An overview of the exhaustive literature survey is provided in Section 2. The methodology adopted is detailed in Section 3, followed by the detailed discussion of obtained results in Section 4. Finally, Section 5 concludes the paper.

## 2. Literature Survey

The resectability assessment is the best accomplished by utilizing the imaging, but the emission tomography positron is unclear [20]. The resectability is the ability of the disease removal while leaving an adequate liver remnant. The routine use of diagnostic laparoscopy is recommended in the patients with high-risk features. The high-risk features of patients should be encouraged and adjuvant therapy is considered. The development of targeted therapeutic interventions is supported by the biliary cancers genomic analyses. The author in this paper details the staging cholangiocarcinoma and determining respectability, for that an accurate noninvasive method which is MRI/MRA/MRCP is detailed [21]. In this paper, the author discussed about the routine lymphadenectomy and defined the positive lymph nodes and predictive indicators of survival in patients. By utilizing the uni- and multivariate analyses, assessment of clinical and pathologic data was done [22]. The patient's age less than 45 having lymph node positive had a 27-month survival. Although prospective data are required, lymph node positive patients have longer survival associated with the adjuvant therapy. For adjuvant therapy, the prognostic information and guidance are provided by the routine lymphadenectomy. In this paper, the author aims to evaluate the patient's outcome, who had delayed staging at 3 months after a cholecystectomy [23]. The preoperative staging using multidetector computed tomography is delayed by the 49 patients who underwent using multidetector computed tomography (MDCT) followed selectively by laparoscopy after a cholecystectomy. The analysis of patient's long-term and perioperative outcomes is performed. The statistical analysis is done by the SPSS tool. A favorable prognosis associated with the intraductal growth (IG) type of intrahepatic cholangiocarcinoma (ICC) is compared with the mass-forming (MF) and periductal-infiltrating (PI) ICC [24]. After controlling for competing risk factors, IG patients had a similar prognosis as MF patients on multivariable analysis. The IG patients' prognosis was comparable with MF patients and the IG patients are frequently presented with adverse pathological characteristics. The author details the lymph node (LN) status which is a survival for resected IHCC [25]. The evaluation of number of LNs resected is done at the time of surgery. The maximal chi-square testing and five-year overall survival were utilized for LN thresholds evaluation. The 3 LNs as the threshold are identified as a maximal chi-square testing. The 39% of resections reached this threshold. The prognostic yield is carefully considered by the surgeons to determine the extended lymphadenectomy at the time of curative-intent resection. Since these tumors vary greatly in location, growth pattern, and histologic type, the radiologic manifestations of cholangiocarcinomas are extremely diverse [7]. For accurate detection and characterization of these tumors and assessment of respectability, the imaging manifestations of cholangiocarcinomas are important. The imaging techniques are advanced and have led to the availability of an array of modalities that is utilized independently. For correct diagnosis and appropriate management of these tumors, the emerging imaging applications are required [26]. The black race was associated with worse survival is demonstrated by the Cox proportional hazard ratio model with worse survival while surgical resection was not independently associated with survival. As compared to chemotherapy alone, the surgical resection for patients with LN-positive ICC may not improve pathologic survival.

## 3. Materials and Methods

The 50 ECC patients (28 males, 22 females; age 45–68), admitted to Indira Gandhi Medical College and Hospital between 2016 and 2019, were selected as research subjects. Inclusion criteria: patients diagnosed with ECC pathologically; patients diagnosed with ECC by imaging examination or tumor markers; patients with abdominal pain, jaundice, or poor appetite or being emaciated; patients with the tumor originating from extrahepatic biliary system.

The principle of DCE-MRI technology: continuous and rapid imaging sequence was used to scan the disease tissue in multiple phases to obtain a series of images at different periods of before, during, and after intravenous injection of contrast agent. The scanning process is shown in Figure 5. The image contains information of tissue perfusion and vascular permeability, and the physiological characteristics of the disease tissue were quantitatively and accurately analyzed based on these parameters [27].

The patients were in the supine position with an empty stomach. The contrast agent gadolinium-diethylenetriaminepentaacetate (Gd-DTPA) was injected intravenously at 0.2 mmoL/kg, with the dynamic enhancement scan starting 15 seconds later.

The patients should hold breath during the whole process. After the contrast agent is injected with a speed of 3 mL/s, another 20 mL normal saline is injected at the same speed to flush the residual contrast agent.

Then, a cross-sectional DCE-MRI examination was performed, with liver acquisition with volume acceleration (LA-VA) scan sequence adopted: repetition time 3.9 ms/echo time 1.9 ms; slice thickness 4.4 mm.

Each scan lasted for 9.3 seconds and there were 35 scans in a row.

All images were reviewed by two doctors with at least 5 years of experience in MRI diagnosis. Those with poor quality and enhancement were excluded. The processed images were analyzed by the o.k software. Three ROIs were selected from the image (away from the vessel and necrotic areas) to measure the Kep, Ve, and Ktrans values, with an average taken from the three.

Pathological classification: according to the Steiner grading system, ECC patients were divided into 3 grades of high differentiation, moderate differentiation, and poor differentiation. If the same pathological tissue had different degrees of differentiation, the dominant differentiation degree was selected as the representative.

Determination of VEGF expression level: immunohistochemical staining method was used to detect the VEGF expression level in ECC patients. To have brown particles in the cytoplasm was considered positive for VEGF expression. Then, the count started, high-power fields were selected to count the number of positive cells and the total number of cells. According to the proportion of positive cells in the tissue, they were divided into 4 levels, as shown in Table 1.

The CD34 was adopted to observe the number of microvessels in the diseased tissue. It was considered positive, if there were brown particles in the vascular endothelial cytoplasm. At first, three areas with the highest vessel density were selected under a low power microscope. Then, the number of stained microvessels in these three areas was counted under a high-power microscope. The average of the three areas was taken as the final result. The data were processed by SPSS 21.0. The measurement data were calculated as mean ± deviation (‾*x* ± *s*). The correlation between ECC perfusion parameters with ECC pathological classification, as well as with VEGF expression, was analyzed by the Spearman test. The Pearson test was for the correlation analysis between ECC and MVD. *P* < 0.05 was set as the threshold for significance.

## 4. Results and Discussion

### 4.1. The DCE-MRI Examination Results

The data used in this work are open access and available publically. There were 15 cases with differentiated carcinoma, 23 cases with moderately differentiated carcinoma, and 12 cases with lowly differentiated carcinoma. Non-VEGF expression was noted in 21 cases, with low expression noted in 15 cases, moderate expression noted in 14 cases, and no high expression case noted. The MVD range was between 40 and 70 among the 50 patients, observed at high power.

### 4.2. The Correlation between the DCE-MRI Perfusion Parameters with Pathological Classification

The Ktrans, Kep, and Ve values of the ECC patients were all not associated with the pathological classification (*P* > 0.05), as shown in Figures 6–8. The correlation between the DCE-MRI perfusion parameters with pathological classification is also given in Table 2.

### 4.3. The Correlation between the DCE-MRI Perfusion Parameters with VEGF Expression

The Ktrans, Kep, and Ve values of the ECC patients were all not associated with the VEGF expression (*P* > 0.05). The correlation between the DCE-MRI perfusion parameters with VEGF expression is shown in Table 3 and graphically presented in Figure 9.

### 4.4. The Correlation between the DCE-MRI Perfusion Parameters with MVD

The MVD of the ECC patients was found to be positively correlated with Ktrans value (*r* = 0.524, *P* < 0.001) and was not associated with the Kep and Ve values, as given in Table 4, and the values are graphically presented in Figure 10.

New vessels are formed mainly based on the existing capillaries in the tissue and venules adjacent to the capillaries. According to the different distribution characteristics of angiogenesis, it can be divided into physiological angiogenesis and pathological angiogenesis [28–31]. The physiological angiogenesis is distributed orderly, and the branches on the main trunk are mostly regular, while the pathological angiogenesis is distributed disorderly and is prone to arteriovenous short circuits. In tumor blood vessels, immature blood vessels with partially missing histological structures account for a large proportion. Due to the lack of a complete basement membrane tightly connected to the cells and a single thin blood vessel wall, the permeability of the tumor blood vessels is greatly improved, resulting in the leakage of substances in the blood vessels. Studies have shown that an increasing number of new blood vessels and the opening of arteriovenous short circuit indicate the further enhancement of tumor tissue invasion and metastasis ability, accompanied by higher malignant degree and pathological classification [32–34].

### 4.5. Comparative Analysis of the Proposed Technique with the Existing Techniques

The proposed technique is compared with the existing technique [10] in terms of *r* value and the ECC perfusion parameters. The comparison is tabulated in Table 5 and also presented graphically in Figure 11 for better analysis and visualization.

It is analyzed and observed from the presented figure that the presented technique is highly correlated than the existing technique. These both techniques are positively correlated with Ktrans value as compared to the Kep and Ve values. The proposed technique performance is evaluated and the improvement in terms of percentage is shown in Figure 12 over the existing technique.

The proposed technique outperforms the existing technique in terms of Ktrans, Kep, and Ve values by 2.75%, 17.37%, and 20.95%, respectively. In this study, the CD34 was used to label ECC blood vessels to count MVD, because its specificity for vascular endothelium is much higher than other markers. The number of tumor neovascularization can be intuitively determined by counting MVD, so as to determine the tumor tissue malignant degree [35]. VEGF is a polypeptide factor that can specifically induce the new blood vessels formation in tumor tissues and usually acts on tumor vascular endothelial cell membranes. Studies have found that there is no correlation between MVD and VEGF. It is because before promoting angiogenesis in pathological tissues, VEGF often needs to go through some complicated processes to act on specific receptors on the vascular endothelial cell membrane [36–38].

MRI is widely used in the current medical imaging by virtue of its multiparameter, multisequence, and multidirectional imaging function. It is a more objective and accurate inspection method. With the continuous development of science and technology, many new magnetic resonance technologies have been developed, such as arterial spin labeling (ASL), diffusion-weighted imaging (DWI), and Perfusion-weighted imaging (PWI). Hence, the MRI has broad development prospects [39].

## 5. Conclusion

The dynamic MR imaging technology can quantitatively reflect the angiogenesis and pathological classification of ECC patients, which has found broad applications in clinical treatment of ECC. However, some limitations should be noted about the technology. At present, the technology cannot be used alone, which is just an assisted method during the conventional MRI examination. MRI is used in the current medical imaging by virtue of its multiparameter, multisequence, and multidirectional imaging function. It is a more objective and accurate inspection method. Further, there is no unified standard when the technology is applied in practice, resulting in lack of reference when an individual image is obtained. The Ktrans, Kep, and Ve values of the ECC patients were all not associated with the pathological classification, with no significant difference (*P* < 0.05). The presented technique is highly correlated than the existing technique. These both techniques are positively correlated with the Ktrans value as compared to the Kep and Ve values. The proposed technique outperforms the existing technique in terms of Ktrans, Kep, and Ve values by 2.75%, 17.37%, and 20.95%, respectively. There is a fixed pharmacokinetic model for the quantitative analysis, whereas some diseased tissues may have interrupted blood supply or multiple blood supply which fails to match the fixed model. In addition, DCE-MRI cannot clearly show the fine blood vessels and blood vessel walls when the vessel area is too large. In the future, with more efforts made in bioengineering, pharmacokinetic models that better match pathological tissues will be established. Furthermore, the imaging speed of dynamic MRI technology will become increasingly faster, and the imaging quality can also be optimized.

## Figures and Tables

**Figure 1:** The classification of cholangiocarcinoma.

**Figure 2:** Intrahepatic cholangiocarcinoma (a) axial T1-weighted and (b) axial T2-weighted.

**Figure 3:** Perihilar cholangiocarcinoma. (a) An MRCP image as a focal stricture and (b) T1W in-phase SGRE; the mass is hypointense relative to liver parenchyma.

**Figure 4:** Intraductal cholangiocarcinoma (a) axial gadolinium-enhanced T1 SGRE image and (b) coronal T2W SSFSE MRCP images.

**Figure 5:** DCE-MRI technology.

**Figure 6:** The Ktrans value of different differentiation grades.

**Figure 7:** The Ve value of different differentiation grades.

**Figure 8:** The Kep value of different differentiation grades.

**Figure 9:** Perfusion parameter with VEGF.

**Figure 10:** Perfusion parameter with MSD.

**Figure 11:** Comparative analysis of the proposed and existing technique.

**Figure 12:** The improvement of the presented technique over existing technique.

**Table 1:** The proportion of positive cells in the tissue.

Positive cells in the tissue			
No positive cell	Positive cell <25%	Positive cell 25%–50%	Positive cell >50%
Unexpressed	Lowly expressed	Moderately expressed	Highly expressed

**Table 2:** The correlation between the DCE-MRI perfusion parameters with pathological classification.

The ECC perfusion parameter	High differentiation (*n* = 15)	Moderate differentiation (*n* = 23)	Low differentiation (*n* = 12)	*r* value	*P* value
Ktrans (min^−1^)	0.431 ± 0.034	0.541 ± 0.161	0.472 ± 0.136	0.124	0.267
Kep (min^−1^)	1.159 ± 0.561	1.521 ± 0.543	1.178 ± 0.965	0.068	0.583
Ve	0.472 ± 0.139	0.463 ± 0.128	0.474 ± 0.232	0.125	0.421

**Table 3:** The correlation between the DCE-MRI perfusion parameters with VEGF expression.

The ECC perfusion parameter	VEGF	
	*r* value	*P* value
Ktrans (min^−1^)	0.024	0.843
Kep (min^−1^)	0.014	0.926
Ve	0.072	0.635

**Table 4:** The correlation between the DCE-MRI perfusion parameters with MVD.

The ECC perfusion parameter	MVD	
	*r* value	*P* value
Ktrans (min^−1^)	0.524	<0.001
Kep (min^−1^)	0.223	0.135
Ve	0.127	0.289

**Table 5:** Comparison of the presented technique with existing technique.

The ECC perfusion parameter	Existing technique (*r* value)	Presented technique (*r* value)
Ktrans (min^−1^)	0.510	0.524
Kep (min^−1^)	0.190	0.223
Ve	0.105	0.127

## Data Availability

All data have been shared in the manuscript.
